The article "Analysis of the Influence of Innovative Teaching Management Mode in Universities on Students' One-to-One Training and Psychotherapy" was retracted in 2023. Reasons: signs of a paper mill; suspected computer-generated content; unreliable results or conclusions; concerns about the data.

# Analysis of the Influence of Innovative Teaching Management Mode in Universities on Students' One-to-One Training and Psychotherapy

**DOI:** 10.1155/2022/8505257

**Published:** 2022-10-12

**Authors:** Wenwen Zhang

**Affiliations:** School of Physical and Mathematical Sciences, Nanjing Tech University, Nanjing, Jiangsu 211816, China

## Abstract

**Objective:**

This study expects to investigate and verify the intervention effect of the university's innovative teaching management model on college students' resilience by implementing the university's innovative teaching management model for college students with low psychological resilience.

**Method:**

The scientific scale is used to investigate the current level of college students' psychological resilience, and the development characteristics of college students' psychological resilience are obtained through statistical analysis. Based on the theoretical analysis of the application of psychological resilience intervention, combined with the theory of one-to-one tutoring and operational techniques, the university's innovative teaching management mode scheme is designed. The design adopts a quasi-experimental pre-experimental test to investigate and explore the intervention effect system of the university's innovative teaching management mode on college students' psychological resilience. In the intervention, each unit of activity is carried out in strict accordance with the established plan, and records and reflections are made at the end. One-to-one and face-to-face qualitative interviews were conducted with the subjects, and qualitative data were collected for qualitative analysis. *Results/Discussion*. Compared with the control group that did not receive the intervention, the psychological resilience of the subjects in the experimental group was significantly improved after receiving the intervention of the university's innovative teaching management model. The university's innovative teaching management model has a good intervention effect on the resilience of college students. The university's innovative teaching management model scheme compiled in this study integrates a variety of psychotherapy methods and combines one-to-one psychological counseling frameworks and techniques. It is an effective and easy-to-implement intervention scheme for college students' psychological resilience intervention.

## 1. Introduction

As a huge systematic project, teaching management activities are faced with the challenges and opportunities presented by the talent quality requirements in the 21st century knowledge economy era [1]. The theory and method of system theory put people-oriented management concept in the first place, carry out the innovation of teaching management concept and the whole process of teaching management, provide a viable soil for the cultivation of innovative talents, and strive to improve the level of management and the quality of teaching and the quality of college students, and gradually adapt to the new teaching management laws [2].

The article "Analysis of the Influence of Innovative Teaching Management Mode in Universities on Students' One-to-One Training and Psychotherapy" was retracted in 2023. Reasons: signs of a paper mill; suspected computer-generated content; unreliable results or conclusions; concerns about the data.

The basic functions and fundamental tasks of colleges and universities are to cultivate talents. Teaching is the regular central work of the school. Teaching management occupies a particularly important position in the management of colleges and universities. It is precisely because the teaching process based on the cultivation of innovative talents has its own particularity that the traditional teaching management model cannot meet the requirements of the cultivation of innovative talents, so reform and innovation must be carried out.

The key to the cultivation of innovative talents is that the school provides college students with a teaching environment that can stimulate their potential and interests, so that college students can become the main body of learning and self-development, gain the right to make independent choices, and have fun in learning and thinking, while teachers change the past and simply impart knowledge [3–5]. Its role is to guide, promote, and encourage college students to study [6–8]. Although the teaching management of colleges and universities is a non-teaching factor, it directly maintains and monitors the teaching of teachers [9]. The main body of teaching management can integrate and control various factors of the teaching environment, extract the factors that have positive significance for the development of the subject, overcome, and eliminate the influence of unfavorable factors, so as to create a teaching environment suitable for the development of innovative talents [10–12]. Good teaching management plays a role in guaranteeing, motivating, and guiding the cultivation of innovative talents.

Teaching management embodies a school's educational ideology and school-running level and is an important aspect of school teaching [13, 14]. Whether the teaching management work is effective or not is directly related to the quality of personnel training. Through the planning, organization, coordination, and control of teaching management, it provides college students with an environment for bold practice, active innovation, and healthy growth, thereby promoting the cultivation of innovative talents [15]. The level of teaching management also affects the training effect and degree of innovative talents [16].

Compared with the control group that did not receive the intervention, the psychological resilience of the subjects in the experimental group was significantly improved after receiving the intervention of the university's innovative teaching management model (*P* < 0.001). The university's innovative teaching management model has a good intervention effect on the resilience of college students.

The article "Analysis of the Influence of Innovative Teaching Management Mode in Universities on Students' One-to-One Training and Psychotherapy" was retracted in 2023. Reasons: signs of a paper mill; suspected computer-generated content; unreliable results or conclusions; concerns about the data.

The university's innovative teaching management model scheme compiled in this study integrates a variety of psychotherapy methods and combines one-to-one psychological counseling frameworks and techniques. It is an effective and easy-to-implement intervention scheme for college students' psychological resilience intervention.

In this university, innovation teaching management model intervention aimed at college students' psychological resilience, intervenor, self-exploration, interpersonal learning, and one-to-one cohesion are all therapeutic factors, and the complex intervention effects of each therapeutic factor on different intervention (protective) factors are combined.

## 2. Methods

### 2.1. The Theoretical Basis of College Teaching Management Reform Based on the Cultivation of Innovative Talents

#### 2.1.1. Management Theory

System science and management are closely related. Any organized management unit has a system, and management is actually the management of a certain system.

The elements are interrelated and form an indivisible whole. Elements are elements in the whole. If the elements are separated from the whole of the system, it will lose the function of the elements. The basic thinking method of system theory is to treat the object to be studied and processed as a system; analyze the structure and function of the system; study the relationship between the system, elements, and the environment and the regularity of changes; and optimize the system point of view.

The principles of system theory are mainly the principle of integrity, the principle of structure and function, the principle of purpose, and the principle of optimization [17, 18]. When the element remains unchanged, the structure determines the function; the principle of purpose, that is, to determine or grasp the system goal and take corresponding means to achieve it, can understand the control in the management process [19].

A university is a social functional system, consisting of a main system (a system that directly undertakes the task of cultivating specialized talents and carries out teaching work), a support system (a system that ensures the work of the main system in terms of manpower, material resources, financial gifts, etc.), and a control system.

The most direct purpose of the teaching management system should be to achieve the maximization of the system gain, and the conditions for obtaining the maximum benefit are determined by the goals, rules, implementation, guarantee, and other factors of the teaching management process.

The article "Analysis of the Influence of Innovative Teaching Management Mode in Universities on Students' One-to-One Training and Psychotherapy" was retracted in 2023. Reasons: signs of a paper mill; suspected computer-generated content; unreliable results or conclusions; concerns about the data.

#### 2.1.2. Business Process Reengineering Theory

The business process reengineering movement aims to significantly improve the performance of an organization, and it emphasizes a fundamental overhaul of traditional management models. Business process reengineering is based on the information network spread across all departments in the organization. It reduces the time loss caused by the flow of information, not only improves the efficiency and reduces the personnel but also enables each employee to have a comprehensive understanding of the overall situation of the enterprise, so that the organization has a new situation.

The teaching management of planning, organizing, leading, and controlling the educational activities of colleges and universities is a very complex systematic process, and its main processes are divided into teaching process, and management process.

#### 2.1.3. People-oriented management theory

Humanistic management theory is the specific application of humanistic psychology in the field of management, which has been popular all over the world. Humanistic theory is based on social and economic development and people's increasing concern and attention to human nature. At first, it was mainly applied to enterprise management. With the development of society, it is more and more applied to other fields of society.

“Basic” has two meanings: one is the fundamental meaning and the other is the meaning of “center, purpose”; as the name suggests, “people-oriented” means people-oriented, people-centered, and people's development as the purpose.

### 2.2. Study Design

This experiment adopts a pre- and post-experimental design. In the experiment, in order to prevent the experimental error caused by the loss of subjects from affecting the experimental results, the experimental group was divided into two groups. Before the start of the experiment, both the experimental group and the control group took a pre-test of psychological resilience. At the end of the last experiment in the eighth week, all the subjects immediately took the post-experiment test and were interviewed within one week after the end of the experiment.

#### 2.2.1. Research Variables

In this study, the independent variable is the university's innovative teaching management model. The experimental group received a 90-minute university innovative teaching management mode once a week for eight weeks. No experimental treatment was performed on the control group during the experimental treatment phase.

The article "Analysis of the Influence of Innovative Teaching Management Mode in Universities on Students' One-to-One Training and Psychotherapy" was retracted in 2023. Reasons: signs of a paper mill; suspected computer-generated content; unreliable results or conclusions; concerns about the data.

The dependent variable is the resilience level score of the subjects measured by the “Adolescent Mental Resilience Scale,” there are five dimension scores and one total score, and the five dimension scores are “target focus” score, “emotion control” score, “positive cognition” score, “interpersonal assistance” score, and “family support” score; the total score is the sum of the scores of the five dimensions, which is the “total psychological resilience score.”

#### 2.2.2. Research Procedures

*(1) Preparatory Stage before the Experiment*. The researchers first checked the relevant literature on resilience and psychotherapy to understand the connotation, structure, theoretical model, and related researches of resilience; to understand the basic conditions and characteristics of adolescent resilience; and to organize and summarize the intervention research on resilience. Secondly, it organizes and summarizes the related researches on the past development, theoretical basis, internal mechanism, and functional effects of psychotherapy and analyzes and records the empirical research of psychotherapy intervention. On this basis, the researchers studied with registered psychotherapists, accepted the supervision of registered psychotherapists, and participated in the practice of psychotherapy to deepen their understanding of psychotherapy interventions. On the basis of the above research, combined with their own thinking and summary, the researcher designed the university innovative teaching management model scheme in this paper and invited registered psychotherapists and psychology professors to review them together, put forward their opinions and make revisions, and finally agreed.

After that, we conduct a questionnaire survey on college students' psychological resilience and screen out the subjects who meet the experimental requirements and invite them to participate in the pre-enrollment interview to ensure that they are willing to participate in the one-to-one training and are willing to abide by the one-to-one training.

*(2) Experimental Intervention Stage*. The 30 subjects in the experimental group were given a 90-minute university innovative teaching management model once a week for eight weeks, and the control group did not receive any experimental treatment. After each one-to-one training, discuss with the assistant actively, and adjust and improve the next one-to-one training plan according to the performance and feedback of the one-to-one training members.

*(3) Post-Experiment Processing Stage*. Immediately after the end of the last one-on-one training, post-test measurements were performed on all experimental group members, and one-on-one, face-to-face qualitative interviews were conducted to obtain more comprehensive quantitative data and qualitative materials. After the data and materials have been collected, statistical analysis of the data will be carried out in a timely manner.

The article "Analysis of the Influence of Innovative Teaching Management Mode in Universities on Students' One-to-One Training and Psychotherapy" was retracted in 2023. Reasons: signs of a paper mill; suspected computer-generated content; unreliable results or conclusions; concerns about the data.

### 2.3. Research Objects

#### 2.3.1. Experimental Subjects

The experimental subjects were all from a certain university. College students with a resilience score lower than one standard deviation from the mean were selected for recruitment. According to the principle of voluntary participation in psychological one-to-one counseling, one-to-one interviews were set up before group enrollment. During the lunch break at noon and within half an hour after school in the afternoon, college students were arranged to participate in the interviews to understand the real wishes and situations of college students.

All subjects were randomly assigned to two experimental groups and one control group according to the principle of gender and grade matching. Considering that the subjects may be lost, the subjects in the experimental group were divided into two treatment groups with equal conditions, with 15 subjects in each group, and 30 subjects in the control group did not receive any experimental treatment.

#### 2.3.2. Researcher

The researcher also serves as the leader of the university's innovative teaching management model in this study, and the leader completes the design of the one-to-one tutoring plan including the collection of literature and the analysis and discussion of the later results. After determining the research topic, the researcher has been studying and practicing with a registered psychotherapist. During this period, he also participated in art psychotherapy seminars and psychotherapy workshops held in China, and he also has a profound experience and perception of psychotherapy. Researchers have received professional psychological one-to-one counseling training during undergraduate and postgraduate studies and have completed more than 100 psychological one-to-one counseling leading and assistant tasks.

### 2.4. Research Tools

In this study, the “Adolescent Mental Resilience Scale” was used for pre-test and post-test.

After the eight-week university innovative teaching management model, all one-to-one members should fill in the form, evaluate the impressions and points of interest of all one-on-one activities, and make their own suggestions. Let the leader understand the feeling of the entire university's innovative teaching management model to the members and use it as an important data for the later qualitative analysis and evaluation of the intervention effect.

The “One-to-One Factor Evaluation Sheet” mainly examines the feelings of one-to-one members on team building factors such as one-to-one cohesion and one-to-one sense of security. It aims to help leaders understand the members' experience and each member's overall perception of the one-to-one situation. The main contents include one-to-one cohesion, one-to-one atmosphere, one-to-one harmony, one-to-one safety, teacher leadership, and overall satisfaction. The scale is incorporated into the “General Feedback Form for the University's Innovative Teaching Management Mode,”, which is filled out by members at the end of the eighth end of the university's innovative teaching management mode.

The article "Analysis of the Influence of Innovative Teaching Management Mode in Universities on Students' One-to-One Training and Psychotherapy" was retracted in 2023. Reasons: signs of a paper mill; suspected computer-generated content; unreliable results or conclusions; concerns about the data.

After the eight-week university innovation teaching management model, a one-on-one interview was conducted with each participant in the experimental group to gain a more comprehensive understanding of the participants' feelings, gains, and thoughts on the university's innovative teaching management model. Interview recordings will serve as an important material for qualitative analysis.

### 2.5. Data Processing

The SPSS 20.0 software package was used for data entry and statistical analysis of the pre- and post-test data.

### 2.6. The Design of the university's Innovative Teaching Management Model

The intervention of psychological resilience generally refers to the intervention of the protective factors of psychological resilience. By strengthening or improving the protective factors in a planned and targeted manner, the psychological resilience of individuals can be effectively improved. Therefore, the design of this program is based on the previous theory of psychological resilience, combined with the “College Student Mental Resilience Scale” to divide the dimensions of college students' psychological resilience, and divided six of the eight one-on-one training activities. The intervention goals of the activity unit are positive self-recognition, good emotional regulation, accurate future planning, effective problem solving, social support-family, and social support-school.

The university's innovative teaching management model scheme in this study was designed based on the theory of one-to-one psychological counseling and Orff's one-to-one music therapy. In Orff one-on-one psychotherapy, the therapist needs to focus on the treatment object and guide the treated person to participate in music activities to the greatest extent in an appropriate way. The design of the activities should fit the physical and mental conditions of the treatment object. In the activity, the performance of the treated person should be affirmed in a timely and appropriate manner, the selection of materials should be as concise as possible, and the therapist should use various types of materials flexibly and fully.

The article "Analysis of the Influence of Innovative Teaching Management Mode in Universities on Students' One-to-One Training and Psychotherapy" was retracted in 2023. Reasons: signs of a paper mill; suspected computer-generated content; unreliable results or conclusions; concerns about the data.

In this study, each unit of the university's innovative teaching management model will be carried out in the procedure of “warm-up game-theme activities-discussion and sharing-summary and extension,” and the stages of each unit are also different. The first unit is the relationship establishment stage. The second to seventh units are the theme implementation stage, and the eighth unit is the one-to-one ending stage.

#### 2.6.1. Relationship Establishment Stage

The purpose of this unit is to make the first-time members familiar with the one-on-one training venue, know the activity time, learn to abide by the rules of the activity, clarify their own one-on-one training goals, try to greet each other with other members, and introduce themselves.

#### 2.6.2. Theme Implementation Stage

The second unit revolves around cultivating members' positive self-awareness. In the music-guided imagination, members can gradually relax with the music, and follow the leader's guiding words to develop rich imagination. The content of the imagination will be drawn in the “Tree of Life” drawing session later, and then everyone will share and discuss.

The goal of the third unit is for members to learn how to listen to the emotional “music” of others, and use music to regulate and control their own emotions. The master will invite a member to play his negative “emotion,” and the master will slowly join in, using music to echo his negative “emotion” music until the member's negative emotions are relieved. Next, invite others to try to do the same and feel the emotional relief.

The goal of Unit 4 is to help members build their dreams, increase their sense of hope, and learn how to plan for achieving their goals. In the “Progressive Relaxation Exercise” session, the members will experience the whole body from tension to relaxation under the leadership of the leader, so that the body is in a relaxed state.

The main purpose of the fifth unit is to improve the members' coping ability in the face of difficulties and adversity, increase the coping style, and learn to deal with it calmly. In the way of group creation of theme songs, let members find difficulties in group cooperation, solve them, and share their experiences afterwards, trigger a “brainstorm” on difficulties and coping methods, and learn more coping methods through discussion.

The sixth unit focuses on the parent-child relationship, mainly to promote members to feel the support from their parents and the good intentions behind them, to experience the difficulties of their parents, and to vent their dissatisfaction. The members discussed the script in small groups, directed the plot, learned the reasons and feelings behind some of their parents' behavior towards them through role-playing, and tapped for more family support.

The article "Analysis of the Influence of Innovative Teaching Management Mode in Universities on Students' One-to-One Training and Psychotherapy" was retracted in 2023. Reasons: signs of a paper mill; suspected computer-generated content; unreliable results or conclusions; concerns about the data.

The goal of Unit 7 is to enhance members' intramural support systems, feel the campus culture by learning and sing the school song, and experience the sense of strength that everyone can overcome all difficulties by working together. In the chorus, members need to coordinate their own voices with others, and they need to learn to cooperate with others or lead everyone. In the process, members can improve their understanding of peer relationships and improve their interpersonal skills. In the following discussion, you can also learn to ask the teacher for help when you encounter difficulties.

#### 2.6.3. One-to-One Ending Stage

The goal of Unit 8 is to help members sort out the gains and feelings of the previous seven activities and deal with the emotions of parting. The leader led the members to review the main activities of each unit before and everyone's insights.

## 3. Results

### 3.1. Comparison of Pre-test Differences between the Experimental Group and the Control Group

The homogeneity test of the psychological resilience pre-test scores of the experimental group and the control group was carried out, and the independent samples *t* test was used for statistics. The results are shown in Figure 1.

It can be seen from Figure 1 that there is no significant difference between the experimental group and the control group before the intervention in the total score of resilience and the pre-test scores in each dimension (*P* > 0.05), indicating that there is no significant difference between the two groups.

### 3.2. Comparison of Pre- and Post-test Differences between the Experimental Group and the Control Group

In order to examine the effectiveness of the intervention of the university's innovative teaching management model, this work takes resilience and its five dimensions as dependent variables. The statistical results are shown in Figure 2.

In the total score of resilience and each dimension, goal focus, emotional control, positive cognition, family support, interpersonal assistance, and total resilience scores have significant interactions between time and group, and emotional control is significant in time and group. The interaction effect is the most significant. It preliminarily shows that the university's innovative teaching management mode has an intervention effect on college students' psychological resilience. The target concentration, emotional control, positive cognition, family support, interpersonal assistance, and psychological resilience of 30 college students are shown in Figure 3. The influence effect test of each index of 30 college students is shown in Figure 4.

The article "Analysis of the Influence of Innovative Teaching Management Mode in Universities on Students' One-to-One Training and Psychotherapy" was retracted in 2023. Reasons: signs of a paper mill; suspected computer-generated content; unreliable results or conclusions; concerns about the data.

### 3.3. One-to-One Factor Evaluation Analysis of University Innovative Teaching Management Mode

The university's innovative teaching management model has a good immediate intervention effect on college students' psychological resilience, but there are still some problems that need to be answered urgently. This research not only collected quantitative data for analysis but also collected some qualitative materials such as feedback sheets and interview recordings. By analyzing the qualitative materials, we can further explain the effect of the intervention and can also explain in a more in-depth and specific manner. In this study, we hope to use qualitative analysis to explain the changes of the experimental group's gains and psychological resilience after accepting the university's innovative teaching management model and to discuss the possible effective therapeutic factors and mechanisms of the university's innovative teaching management model.

After the eight-week university innovative teaching management model ended, all one-to-one members made subjective evaluations on one-to-one factors such as one-to-one cohesion and one-to-one security. The specific results are shown in Table 1.

As can be seen from Table 1, after eight weeks of the university's innovative teaching management model, all one-on-one members feel better in terms of team factor. The one-to-one members have a good feeling about the innovative teaching management model of the whole university. Whether it is the theme setting of each unit or the unit activities, they are welcomed by the one-to-one members, and each member has a certain harvest and growth. The factors ranked from low to high are cohesion, harmony, atmosphere, safety, and teacher leadership. Among the factors, the evaluation of teacher leadership is the highest, indicating that the behavior of the leader in leading the university to innovate the teaching management model has been recognized by the subjects.

In the future, the leader should be good at using the accumulated experience and good practices when holding the university's innovative teaching management model in the future and strive to establish a good dynamic relationship with one-to-one members faster and better. In addition, the evaluation of one-to-one safety and one-to-one atmosphere is also high, indicating that in the university's innovative teaching management model, members and leaders create a safe atmosphere together. Such an atmosphere is conducive to members opening their hearts at ease, sharing their true feelings and insights, and also helping to achieve deeper self-exploration.

The article "Analysis of the Influence of Innovative Teaching Management Mode in Universities on Students' One-to-One Training and Psychotherapy" was retracted in 2023. Reasons: signs of a paper mill; suspected computer-generated content; unreliable results or conclusions; concerns about the data.

### 3.4. Analysis of the Intervention Effect of the university's Innovative Teaching Management Model

In order to examine the intervention effect of the university's innovative teaching management model, the researchers used the interview method to conduct structured interviews with the subjects in the experimental group. After converting the interview recordings into texts, they were coded with reference to grounded theory.

After the initial encoding is completed, focus encoding is performed to inductively combine similar encodings. After the focus coding is completed, it is necessary to develop core categories, and continuously condense the coded content, and finally form a positive self and difficult cognition. There are five categories of interpersonal support. The overall situation of psychological resilience is shown in Table 2.

## 4. Discussion

### 4.1. Teaching Management System: A Booster for the Cultivation of Innovative Talents

In terms of its source, the teaching management system of colleges and universities can be divided into two types: one is the laws and regulations, documents, outlines, etc., of the national education administrative organs to manage teaching [20–22].

The current teaching management system is not conducive to the development of college students' creative personality [23–25]. It is based on the traditional elite education system and is a product of the planned economy. It has played a positive role in stabilizing the normal teaching order of the university and ensuring the teaching quality [26].

The student status management system imposes more restrictions on college students when they exercise their rights to choose majors, study years, study content, and study methods, thus affecting the implementation effect of the elective system and credit system in colleges and universities [27].

The serious power tendencies of the current teaching management organizations lead to unequal teaching management systems [28]. In the teaching management system, teachers and students are placed in the position of objects to be managed [29]. College students cannot effectively and actively exercise the right to participate in teaching management and teaching activities if they cannot understand the school's rules and regulations and development direction, and know and supervise the school or department's exercise of activities related to the interests of college students, which is not conducive to them [30].

### 4.2. Innovation of Teaching Management Methods Based on Creative Development of College Students

Using the theory of process reengineering, the original highly centralized power is shifted downward, and the teaching management functions are decentralized to implement vertical power structure adjustment [31]. The “school-college-department (teaching and research office)” three-level organizational and secondary management model is actually to clarify the responsibilities and powers between the Academic Affairs Office of the higher education institution and the secondary colleges, appropriately carry out hierarchical teaching management, and appropriately expand the secondary colleges [32]. Management authority, the management of secondary colleges by the school's academic affairs office, has changed from “strengthening process management” to “strengthening target management,” activating the school's school-running mechanism and improving the school's management efficiency [33].

The article "Analysis of the Influence of Innovative Teaching Management Mode in Universities on Students' One-to-One Training and Psychotherapy" was retracted in 2023. Reasons: signs of a paper mill; suspected computer-generated content; unreliable results or conclusions; concerns about the data.

The situation of each department is different, and the requirements are also different. The department lacks autonomy, and its main role cannot be fully exerted, which seriously affects the cultivation of innovative talents. In fact, the Academic Affairs Office of the school is not capable of solving all problems related to teaching, and the faculties and departments are the teaching units that directly face the front line of teaching. Only by decentralizing power, properly decentralizing, and establishing a “school-college-department” three-level organizational and two-level management model for teaching management can we better promote the cultivation of innovative talents.

The Academic Affairs Office of the school works under the leadership of the vice-principal in charge of teaching. It is the functional department of the school to manage the teaching work. It plays its decision-making role in the teaching management work and performs the functions of macrocontrol and target management in the teaching work of the whole school [34]. The overall coordination and scheduling of the teaching management work of the colleges and universities, and the provision of guidance and services to achieve the goals of efficient, high-quality, and orderly teaching management [35].

The department (teaching and research section) implements the teaching plan. Its main responsibilities are to implement the teaching plan, carry out education and teaching research, carry out various teaching methods and teaching methods reform, and carry out curriculum construction, teaching material construction, and teaching syllabus according to the planning goals of the college [36, 37].

The teaching process is only forced to be managed by teachers or administrative departments, which will only suppress the enthusiasm of college students. The purpose of teaching management is not to make educational objects obey certain rules unconditionally but to encourage educational objects to accept rational self-direction and self-determination. Allowing college students to participate in management can make college students understand the necessity of teaching management and obey the management. On the other hand, it can give full play to its potential, analyze the ways and methods of each link of teaching management, and truly make college students manage themselves.

The article "Analysis of the Influence of Innovative Teaching Management Mode in Universities on Students' One-to-One Training and Psychotherapy" was retracted in 2023. Reasons: signs of a paper mill; suspected computer-generated content; unreliable results or conclusions; concerns about the data.

### 4.3. Modern Teaching Information Management Model Innovation

The means of teaching management is a yardstick for measuring the level of a school's teaching management. The innovation of teaching management means is one of the main contents of teaching management innovation, and colleges and universities are places for cultivating senior professional talents for the society.

Colleges and universities should become representatives of advanced culture, advanced technology, and advanced management. Only under the education and influence of this atmosphere can college students learn to make full use of advanced technology to continuously improve themselves and cultivate them into talents who stand at the forefront of the times.

Implementing the modernization and informatization of teaching management methods can liberate teaching managers from trivial matters such as the collection, processing, and updating of a large amount of information and data, thereby improving the work efficiency and work quality of teaching management [17, 38, 39].

In the teaching management information system, teaching administrators can set access rights control, information update, function maintenance, and other operations and check the total data provided by secondary colleges [40].

College students can also submit online classroom teaching quality evaluation, tutor evaluation, practice, practice evaluation, textbook evaluation, etc., so that teaching quality information can be timely feedback, which is conducive to the monitoring of teaching quality.

Through the system message function, teachers and students can reflect their various ideas, opinions, and suggestions related to teaching management to teaching managers, which is conducive to timely feedback and exchange of various teaching management information. Thus, teaching managers can better understand the needs of students and teachers and better serve students and teachers.

### 4.4. Discussion on the Effect of Immediate Intervention

From the quantitative analysis results, the two groups of participants are homogeneous before receiving the intervention [41–43]. After the intervention, two-factor repeated-measures variance analysis was performed on the pre-test and post-test data of the two groups [28, 44, 45].

The article "Analysis of the Influence of Innovative Teaching Management Mode in Universities on Students' One-to-One Training and Psychotherapy" was retracted in 2023. Reasons: signs of a paper mill; suspected computer-generated content; unreliable results or conclusions; concerns about the data.

Further analysis of the effect of group and time on the intervention effect is carried out [46–48]. In the simple effect test of time, the total score of psychological resilience of the experimental group and the control group was significantly different from each dimension in the post-test, and the total psychological resilience of the experimental group was significantly different [49, 50].

After the musical sound is received by the body's auditory organs, it is perceived by the brain in a unique emotional form [51]. Let members associate music with emotions and regulate their own or other people's “emotions” in the subsequent “emotional dialogue.” After such exercises, members' understanding, perception, and control of emotions will become more obvious [52, 53].

## 5. Conclusion

There was no significant difference in the level of psychological resilience between the experimental group and the control group before receiving the intervention of the university's innovative teaching management model; that is, the two groups of participants were homogeneous before receiving the intervention. After the intervention, two-factor repeated-measures variance analysis was performed on the pre-test and post-test data of the two groups. Further analysis of the effect of group and time on the intervention effect is carried out. When randomizing the experimental group and the control group, the gender distribution was also relatively uniform. The difference in being better than females minimized interference with the experimental results. These measures in subject selection not only ensure the homogeneity of the research objects but also improve the external validity, and the improvement of the psychological control dimension also suffers less irrelevant effects.

## Figures and Tables

**Figure 1:** The difference test of psychological resilience between the experimental group and the control group (pre-test).

**Figure 2:** Analysis of variance before and after the experimental group and the control group.

**Figure 3:** The goal focus, emotional control, positive cognition, family support, interpersonal assistance, and resilience of 30 college students.

**Figure 4:** The influence effect test of each index of 30 college students.

**Table 1:** Factor evaluation and analysis of one-to-one training in psychotherapy.

Factor	Cohesion	Safety	Atmosphere	Overall satisfaction	Teacher leadership	Harmony
M	7.8	8.4	8.1	7.9	8.5	8.7
SD	1.7	2.4	1.9	2.1	1.8	2.3

**Table 2:** Overall situation of psychological resilience.

Project	Goal focus	Emotional control	Positive cognition	Family support	Interpersonal assistance	Total resilience score
Minimum	4	7	5	6	3	27
Maximum	32	37	28	34	29	124
*M*	17	19	24	21	18	96
Item mean	3.2	3.4	3.8	3.1	2.9	3.3

The article "Analysis of the Influence of Innovative Teaching Management Mode in Universities on Students' One-to-One Training and Psychotherapy" was retracted in 2023. Reasons: signs of a paper mill; suspected computer-generated content; unreliable results or conclusions; concerns about the data.

## Data Availability

The data used to support the findings of this study are available from the corresponding author upon request.
